# An Efficient Algorithm for the Detection of Outliers in Mislabeled Omics Data

**DOI:** 10.1155/2021/9436582

**Published:** 2021-12-22

**Authors:** Hongwei Sun, Jiu Wang, Zhongwen Zhang, Naibao Hu, Tong Wang

**Affiliations:** ^1^Department of Health Statistics, School of Public Health and Management, Binzhou Medical University, Yantai City, Shandong 264003, China; ^2^Department of Health Statistics, School of Public Health, Shanxi Medical University, Taiyuan City, Shanxi 030001, China

## Abstract

High dimensionality and noise have made it difficult to detect related biomarkers in omics data. Through previous study, penalized maximum trimmed likelihood estimation is effective in identifying mislabeled samples in high-dimensional data with mislabeled error. However, the algorithm commonly used in these studies is the concentration step (C-step), and the C-step algorithm that is applied to robust penalized regression does not ensure that the criterion function is gradually optimized iteratively, because the regularized parameters change during the iteration. This makes the C-step algorithm runs very slowly, especially when dealing with high-dimensional omics data. The AR-Cstep (C-step combined with an acceptance-rejection scheme) algorithm is proposed. In simulation experiments, the AR-Cstep algorithm converged faster (the average computation time was only 2% of that of the C-step algorithm) and was more accurate in terms of variable selection and outlier identification than the C-step algorithm. The two algorithms were further compared on triple negative breast cancer (TNBC) RNA-seq data. AR-Cstep can solve the problem of the C-step not converging and ensures that the iterative process is in the direction that improves criterion function. As an improvement of the C-step algorithm, the AR-Cstep algorithm can be extended to other robust models with regularized parameters.

## 1. Introduction

The first challenge presented by omics data is the high dimension, which far exceeds the sample size. The second challenge is the presence of noise in the omics data. This noise may be caused by misdiagnosis, mislabelling, recording errors, technical problems in the laboratory, or sample heterogeneity [1, 2]. Penalized regression is a common method to solve the problem of variable selection and prediction for a high-dimensional dataset. It has been applied to omics data such as gene expression (4), GWAS [3], and DNA methylation [4]. However, the outliers in the data make the estimation of penalized regression inaccurate, so biomarkers cannot be properly screened. Additionally, the identification and further investigation of these outliers can correct the errors during the experiment or investigation. Therefore, it is very important to develop robust statistical methods for penalized regression.

A robust estimation method, least trimmed square (LTS), was proposed by Rousseeuw [5]. LTS is highly robust to outliers in both the response and predictors. It is effective for identifying outliers and can solve the problem of the masking phenomenon caused by the coexistence of multiple outliers [5, 6]. Alfons et al. [6] applied LTS to LASSO-type penalized linear regression to solve the problem of robust high-dimensional variable selection when the dependent variable is quantitative data. Kurnaz et al. [7] applied LTS to elastic net- (EN-) type penalized linear and logistic regression to solve the problem of robust high-dimensional variable selection when the dependent variable is quantitative and binary data (enetLTS).

Both studies adopted the concentration step (C-step) in the FAST-LTS algorithm proposed by Rousseeuw and Van Driessen [8]. The basic ideas were an inequality involving order statistics and sums of squared residuals. This inequality guarantees that the criterion function declines monotonically as the iteration progresses. However, when it is applied to penalized regression based on trimming, the inequality does not necessarily hold due to the change of the regularized parameters. Thus, the criterion function cannot be guaranteed to decrease. Through our previous simulation study [9], we have found that enetLTS is effective in identifying mislabeled samples in high-dimensional data with mislabeled error. However, it is also found that for a dataset with *n* = 500, *p* = 1,000, and an outlier ratio of 10%, it takes nearly 2 hours (Intel Core i7-6500U @2.50GHz) to run enetLTS once. For the omics data in real data analysis with *n* = 924 and *p* = 19690, enetLTS running time is about 77.8 hours (Intel Xeon Silver 4112 @2.60GHZ), which obviously does not meet the requirements for efficient data processing.

Therefore, the C-step algorithm needs to be improved to adapt to high-dimensional data. In this study, the AR-Cstep algorithm is proposed to solve the estimation of robust penalized regression based on trimming, which combines the C-step algorithm with the acceptance-rejection algorithm proposed by Chakraborty and Chaudhuri [10] . Two algorithms are compared in terms of variable selection and outlier identification accuracy and computation speed in simulation study. An RNA-seq dataset for triple negative breast cancer (TNBC) [1] that contains 28 samples with discordant labels obtained from different tests (immunohistochemical (IHC) method or fluorescence in situ hybridization (FISH)) is used to illustrate the application of the two algorithms.

The structure of this paper is as follows: In results section, simulation experiments are described that compare the MTL-EN (elastic net-type maximum trimmed likelihood) estimation using the AR-Cstep algorithm with enetLTS. The results of enetLTS and MTL-EN applied to a triple negative breast cancer (TNBC) RNA-seq dataset are compared. Then, the results are discussed and concluded.

In this article, a robust penalized logistic regression model based on trimming is introduced in Section 2. And the AR-Cstep algorithm is proposed and described in Section 3. In Section 4, simulation experiments are described that compare the MTL-EN (elastic net-type maximum trimmed likelihood) estimation using the AR-Cstep algorithm with enetLTS. The results of enetLTS and MTL-EN applied to a triple negative breast cancer (TNBC) RNA-seq dataset are compared in Section 5. We conclude with a discussion in Section 6 and a conclusion in Section 7.

## 2. Robust Penalized Logistic Regression Model Based on Trimming

Kurnaz et al. [7] proposed an EN-type penalized logistic regression based on trimming.

(1) $$\begin{array}{c} {\overset{\wedge }{\beta }}^{\text{enetLTS}}={\text{argmin}}_{\beta }\overset{h}{\underset{l=1}{\sum }}d\left(y_{i_{l}},x_{i_{l}}^{\prime }\beta \right)+h\lambda P_{\alpha }\left(\beta \right), \end{array}$$

where *d*(*y*_*i*_1__, *x*_*i*_1__′**β**) ≤ *d*(*y*_*i*_2__, *x*_*i*_2__′**β**) ≤ ⋯≤*d*(*y*_*i*_*n*__, *x*_*i*_*n*__′**β**),  *i*_*l*_ ∈ {1, 2, ⋯, *n*}, where d(*y*_*i*_*k*__, *x*_*i*_*k*__′**β**) is the ordered deviance. *h* = ⌊*δn*⌋ (⌊.⌋ means rounding down to the nearest integer) and *α* ∈ [0.5,1], where 1 − *δ* is the trimmed portion. Compared with EN, enetLTS only retains *h* observations with the smallest deviances, whereas *n*-*h* least likely observations under the given model are excluded.

Robust penalized logistic regression model based on trimming was denoted as enetLTS (robust EN based on the LTS), and C-step algorithm was adopted. We denote it as ${\overset{\wedge }{\beta }}^{\text{enetLTS}}$ in this paper. The estimate of the same model obtained by the AR-Cstep algorithm is recorded as the EN-type maximum trimmed likelihood estimate ${\overset{\wedge }{\beta }}^{MTL-EN}$.

## 3. Algorithm

### 3.1. C-Step Algorithm

Kurnaz et al. [7] adopted the C-step algorithm in enetLTS. This algorithm was described below.

Let *Q*(*H*; **β**) be the criterion function of the penalized logistic regression based on the subsample *H*⊆{1, 2, ⋯, *n*}, where |*H*| = *h*. Thus,

(2) $$\begin{array}{c} Q\left(H;\beta \right)=\underset{i\in H}{\sum }d\left(y_{i},x_{i}^{\prime }\beta \right)+h\overset{p}{\underset{j=1}{\sum }}\lambda \left|\beta_{j}\right|. \end{array}$$

Additionally, ${\hat{\;\beta }}_{H}$ represents ${\hat{\;\beta }}_{H}=\arg\underset{\beta }{\min}Q\left(H,\beta \right)$.

When the regularized parameters *λ* = *λ*_1_ and *α* = *α*_1_ are fixed, at the *k*th step of the iteration, *H*_*k*_ is the current subset with *h* observations, and ${\hat{\beta }}_{H_{k}}$ is the solution of the penalized logistic regression based on *H*_*k*_. The negative log-likelihood functions corresponding to *n* observations can be derived from ${\hat{\beta }}_{H_{k}}$. The subsample *H*_*k*+1_ consists of the *h* smallest negative log-likelihood observations, that is,

(3) $$\begin{array}{c} H_{k+1}=\left\{i_{1},i_{2}\cdots ,i_{h}\right\}, \end{array}$$

where $d\left(y_{i_{1}},x_{i_{1}}^{\prime }{\hat{\beta }}_{H_{k}}\right)\leq d\left(y_{i_{2}},x_{i_{2}}^{\prime }{\hat{\beta }}_{H_{k}}\right)\leq \cdots \leq d\left(y_{i_{n}},x_{i_{n}}^{\prime }{\hat{\beta }}_{H_{k}}\right)$, *i*_*l*_ ∈ {1, 2, ⋯, *n*}.

Thus, $Q\left(H_{k+1};{\hat{\beta }}_{H_{k}}\right)\leq Q\left(H_{k};{\hat{\beta }}_{H_{k}}\right)$ can be obtained. *H*_*k*+1_ is the subset that minimizes the criterion function under the solution ${\hat{\beta }}_{H_{k}}$. Then, penalized logistic regression is applied to subset *H*_*k*+1_. If *λ* = *λ*_1_ and *α* = *α*_1_ are unchanged, we get the solution ${\hat{\beta }}_{H_{k+1}}$ which minimize the solution of criterion function under the regularization parameters *λ*_1_ and *α*_1_. Thus $Q\left(H_{k+1};{\hat{\beta }}_{H_{k+1}}\right)\leq Q\left(H_{k+1};{\hat{\beta }}_{H_{k}}\right)$ holds. Therefore, when *λ* = *λ*_1_ is fixed,

(4) $$\begin{array}{c} Q\left(H_{k};{\hat{\beta }}_{H_{k}}\right)\geq Q\left(H_{k+1};{\hat{\beta }}_{H_{k}}\right)\geq Q\left(H_{k+1};{\hat{\beta }}_{H_{k+1}}\right). \end{array}$$

The definition of *H*_*k*+1_ makes the first equation hold. The definition of ${\hat{\beta }}_{H_{k+1}}$ makes the second inequality hold.

For the C-step algorithm, the candidate subset *H*_*k*+2_ is constructed by sorting out *h* samples with the smallest negative log-likelihood contribution to $Q\left(H_{k+1};{\hat{\beta }}_{H_{k+1}}\right)$. Then, the C-step algorithm continues until  *Q*_*m*_ = *Q*_*m*−1_.

Therefore, when *λ* = *λ*_1_ and *α* = *α*_1_ remain unchanged, as the number of iterations *k* increases, the criterion function decreases. Because the criterion function is nonnegative and the number of subsets with sample size *h* is limited, the C-step algorithm must converge to the subset with the smallest criterion function after a limited number of steps.

The C-step algorithm is described in Algorithm 1, where “continueCstep” is set so that the absolute value of the difference between the likelihood functions of two iterations is less than some small value.

However, when penalized regression is performed on the subset *H*_*k*+1_, the regularized parameters *λ* and *α* are not fixed. The regularized parameters are usually determined by data, such as by cross-validation. The regularized parameters determined for penalized regression performed on two different subsets are often different, which leads to the second inequality of [11] not necessarily being true.

A way to solve the problem is to set all *λ* and *α* values firstly. For a certain combination of *λ* and *α*, perform the C-step algorithm until convergence. Then, compare the convergent subsets under different regularized parameters, and select the subset that minimizes the criterion function. If the number of *λ* values is 40 and that of *α* values is 20, there are 800 parameter combinations. This means running the C-step algorithm 800 times, which will undoubtedly make the algorithm very slow.

### 3.2. AR-Cstep Algorithm

In this study, the AR-Cstep algorithm is proposed to solve the estimation of the robust penalized regression based on trimming, which combines the C-step algorithm with the acceptance-rejection algorithm, which was proposed by Chakraborty and Chaudhuri [10].

#### 3.2.1. Acceptance-Rejection Algorithm

The acceptance-rejection algorithm is similar to that of Metropolise-Hastings in MCMC. Let *H*_*k*_ represent the subset at the *k*th step of the iteration. Then, a randomly selected sample outside of *H*_*k*_ replaces one of the samples in *H*_*k*_ to form *H*_cand_. The corresponding likelihood function is obtained after penalized regression is performed on *H*_cand_. If the criterion function corresponding to *H*_cand_ is better than that corresponding to the current subset *H*_*k*_, then *H*_cand_ is accepted as *H*_*k*+1_ with probability one, and *H*_*k*+1_ = *H*_cand_. Otherwise, *H*_cand_ is accepted as *H*_*k*+1_ with a probability of *p* < 1, so that the algorithm can escape the local optimal value.

In the acceptance-rejection algorithm, the candidate sample at each step is randomly selected from the remaining samples other than the current subset *H*_*k*_. Thus, whether the candidate subset can improve the criterion function better is completely random, which leads to the slower convergence of the iteration. The advantage of this algorithm is that, whether the criterion function corresponding to the candidate subset is better than that of the current subset is examined at each step. Moreover, the subset with the optimal criterion function up to the current step is recorded at each step.

#### 3.2.2. AR-Cstep Algorithm

The changes of the regularized parameters *λ* and *α* make the C-step algorithm hardly gradually converge to the subset with the smallest criterion function. Suppose the current subset is *H*_*k*_, and we obtain ${\hat{\beta }}_{H_{k}}$, and corresponding criterion function $Q\left(H_{k};{\hat{\beta }}_{H_{k}};\lambda_{1},\alpha_{1}\right)$ after the penalized regression is performed on *H*_*k*_. The *h* smallest negative log-likelihood observations constitute the subset *H*_cand_, so that $Q\left(H_{\text{cand}};{\hat{\beta }}_{H_{k}};\lambda_{1},\alpha_{1}\right)\leq Q\left(H_{k};{\hat{\beta }}_{H_{k}};\lambda_{1},\alpha_{1}\right)$ holds. Then, penalized regression is performed on *H*_cand_, ${\hat{\beta }}_{H_{\text{cand}}}$ is obtained, and the corresponding regularized parameters changed to *λ*_2_ and *α*_2_. The corresponding criterion function $Q\left(H_{\text{cand}};{\hat{\beta }}_{H_{\text{cand}}};\lambda_{2},\alpha_{2}\right)$ of *H*_cand_ is not necessarily less than $Q\left(H_{\text{cand}};{\hat{\beta }}_{H_{k}};\lambda_{1},\alpha_{1}\right)$. The AR-Cstep algorithm adds the step of comparing the criterion function of the candidate subset *H*_cand_ with that of the current subset *H*_*k*_. If $Q\left(H_{\text{cand}};{\hat{\beta }}_{H_{\text{cand}}};\lambda_{2},\alpha_{2}\right)>Q\left(H_{k};{\hat{\beta }}_{H_{k}};\lambda_{1},\alpha_{1}\right)$, to avoid falling into a local optimum, *U* is a random number that follows the Bernoulli distribution with *p*, where $p=e^{\tau_{k}\left(\log\ell \left({\overset{\wedge }{\beta }}_{H_{\text{cand}},}H_{\text{cand}}\right)-\log\ell \left({\overset{\wedge }{\beta }}_{H_{k},}H_{k}\right)\right)}$. If *U* = 1, then *H*_*k*+1_ = *H*_cand_. If *U* = 0, then *H*_*k*+1_ = *H*_*k*_, that is, no replacement. The criterion function corresponding to the initial subset is recorded as the optimal subset, that is, $Q\left(H_{\text{opt}};{\hat{\beta }}_{H_{\text{opt}}}\right)=Q\left(H_{0};{\hat{\beta }}_{H_{0}}\right)$, and *H*_opt_ = *H*_0_. At each step of the iteration, the criterion function $Q\left(H_{k};{\hat{\beta }}_{H_{k}}\right)$ is compared with $Q\left(H_{\text{opt}};{\hat{\beta }}_{H_{\text{opt}}}\right)$. If $Q\left(H_{k};{\hat{\beta }}_{H_{k}}\right)<Q\left(H_{\text{opt}};{\hat{\beta }}_{H_{opt}}\right)$, then $Q\left(H_{\text{opt}};{\hat{\beta }}_{H_{opt}}\right)=Q\left(H_{k};{\hat{\beta }}_{H_{kt}}\right)$ and *H*_opt_ = *H*_*k*_. *H*_opt_ in the last step is the solution.

To make the proportion of samples with *y* = 1 in the candidate subset *H*_cand_ consistent with that in the full set, the samples constituting the candidate subset *H*_cand_ are selected in the following manner. *H*_cand_ consists of *h*_1_ observations with the smallest $d\left(y_{i},x_{i}^{\prime }{\hat{\beta }}_{H_{k}}\right)$ among observations with *y* = 1 (set a total of *n*_1_ observations), and *h*_0_ observations with the smallest $d\left(y_{i},x_{i}^{\prime }{\hat{\beta }}_{H_{k}}\right)$ among observations with *y* = 0 (set a total of *n*_0_ observations), where *h*_1_ = ⌊(*n*_1_ + 1)*η*⌋, and ⌊.⌋ means round down. 1 − *η* is the trimming ratio and *h*_0_ = *h* − *h*_1_. In comparison with the acceptance-rejection algorithm, for which *H*_cand_ consists of samples selected randomly from the complementary set, *H*_cand_ of AR-Cstep is composed of observations with the smallest deviance; that is, each sample of *H*_cand_ contains information that improves the criterion function; hence, the algorithm converges to the subset with the optimal criterion function faster. The AR-Cstep algorithm is described in Algorithm 2.

The acceptance probability $p=e^{\tau_{k}\left(\log\ell \left({\overset{\wedge }{\beta }}_{H_{\text{cand}},}H_{\text{cand}}\right)-\log\ell \left({\overset{\wedge }{\beta }}_{H_{k},}H_{k}\right)\right)}$. It is inversely proportional to the absolute value of the difference between the two likelihood functions $\log\ell \left({\hat{\beta }}_{H_{k},}H_{k}\right)$ and $\log\ell \left({\hat{\beta }}_{H_{\text{cand}},}H_{\text{cand}}\right)$. The acceptance probability *p* is also related to *τ*_*k*_. According to *τ*_*k*_≔log(*k* + 1)/*D*, the acceptance probability *p* is inversely proportional to *k*, which is the *k*th step of the iteration. Similar to the study of Farcomeni and Viviani [12], *D*≔0.1*n*(1 − *η*), and the acceptance probability *p* is inversely proportional to the sample size *h* of the subset. When other features remain unchanged, the larger the sample size *h* of the subset, the smaller the probability of being accepted. Additionally, if the current subset is not replaced after *r* iterations, the iteration process is stopped.

To ensure that the initial subset does not contain outliers, the sample size should be smaller. The initial subset consisted of six observations, three of which were randomly selected from groups *y* = 1 and *y* = 0, respectively. In order to make the algorithm reach the global optimal value, multiple initial subsets were selected.

First, the two-step iteration of AR-Cstep was performed on 500 initial subsets, and 500 updated subsets were obtained. Then, the 10 subsets with the smallest criterion function were retained. Then, AR-Cstep was performed on these 10 subsets until convergence. Among the 10 convergent subsets, the subset with the smallest criterion function was selected, denoted by *H*_opt_. The penalized regression was performed on *H*_opt_, and ${\hat{\beta }}_{\text{opt}}$ was obtained.

#### 3.2.3. Reweighted Step

In this article, we choose the subset of size *h* = ⌊*nη*⌋ where *η* = 0.75. So 1 − *η* is the initial guess that less than 25% of outliers contained in the data. This is a rather conservative estimation of proportion of outliers. There may not be so many outliers in the data. Therefore, reweighted step is considered to detect outliers via ${\hat{\beta }}_{\text{opt}}$. Then, these outliers are excluded, and a new subset  *H*_rwt_ is obtained. Then, EN-type penalized logistic regression is applied to  *H*_*rwt*_ to get the solution ${\hat{\;\beta }}_{rwt}$. Usually, the size of  *H*_*rwt*_ is larger than *h*, such that more samples can improve the performance of ${\hat{\;\beta }}_{rwt}$ compared to ${\hat{\beta }}_{\text{opt}}$. We called ${\hat{\;\beta }}_{rwt}$ reweighted MTL-EN (Rwt MTL-EN). To distinguish them, the unweighted ${\hat{\beta }}_{opt}$ is called Raw MTL-EN.

#### 3.2.4. Choice of the Regularized Parameters and Standardization of Predictors

We select *λ* over a grid of values in the interval (0, *λ*_max_] as discussed by Breheny and Huang [13].

(5) $$\begin{array}{c} {\hat{\lambda }}_{\max}=\underset{j\in \left\{1,2,\cdots ,p\right\}}{\max}n^{-1}X_{j}^{\prime }y, \end{array}$$

where **y** is the dependent variable and **X**_*j*_ is the *j*th independent variable. In iteration step of AR-Cstep, we take a grid with steps of size 0.05 ${\hat{\lambda }}_{\max}$ and *α* = 0.5 to reduce the computational burden. In the reweighted step, we take a grid with steps of size 0.01 ${\hat{\lambda }}_{\max}$ of *λ* to derive the solution ${\hat{\beta }}_{\text{opt}}\text{ and }{\hat{\;\beta }}_{rwt}$. The choice of *α* is selected by cross-validation in the interval [0.1,1] with a step size of 0.1.

It would be better to standardize predictors before applying the penalized regression. Standardization mainly is aimed at eliminating the influence of dimension and quantity of a predictor. However, the mean and standard deviation computed from all sample are not robust with outliers. In the algorithm described above, penalized regression is applied to the subset in every iteration step of AR-Cstep. So we firstly, respectively, compute mean and standard deviation from subsamples. Then, we standardize all samples with this mean and standard deviation before applying penalized regression.

## 4. Simulation Study

### 4.1. Comparison of MTL-EN and enetLTS on Outlier Detection and Variable Selection

Simulation settings were the same as Sun et al. [9]. The parameter *h* of both enetLTS and MTL-EN was both set to ⌊0.75*n*⌋, which meant the trimmed rate is 25%. The parameters in Ensemble followed Lopes et al. [1].

In the simulation experiment, we compared the two methods enetLTS and MTL-EN using C-step and AR-Cstep algorithms, respectively. Through our previous research [9] and subsequent simulation experiments, we can see that enetLTS is good at identifying outliers. However, the FDR of its variable selection is high, and many unrelated variables are identified. When encountering mislabeled omics data, we can combine enetLTS with Ensemble. Running Ensemble on a subset of data after removing the outliers identified by enetLTS improved the variable selection accuracy. Then, we added the third method Ensemble to the simulation experiment. A detailed description of Ensemble is provided in our previous study [9].

The performances of the three methods are summarized in Figure 1.

The outlier detection accuracy of the three methods is shown in Figure 1. Here, we used two indicators Sn (sensitivity) and FPR (False Positive Rate) [14]. Sn represents the proportion of true misclassified individuals identified as misclassified ones among all true misclassified observations. FPR represents the proportion of individuals with correct labels that are wrongly categorized as misclassified ones.

The outliers identified by MTL-EN had the higher Sn than enetLTS. When the proportion of outliers were 10% and 15%, the gap between them further widened. MTL-EN FPRs were close to enetLTS. Ensemble has the lowest Sn and FPRs among the three methods. Therefore, MTL-EN had the best accuracy in identifying outliers.

The variable selection accuracy of the three methods is shown in Figure 1. PSR (Positive Selection Rate) indicates the proportion of true disease-related biomarkers identified in all true disease-related biomarkers. FDR (False Discovery Rate) represents the proportion of biomarkers that are not related to disease among all the screened biomarkers. A comprehensive indicator GM [15, 16] for the accuracy of variable selection was used, which is the geometric mean of PSR and (1 − FDR). High accuracy of variable selection is indicated by a high GM.

MTL-EN variable selection accuracy was very similar to enetLTS with high PSR and FDR. As also shown in our previous study [9], Ensemble had the highest variable selection accuracy with much low FDR; however, Ensemble missed some associated variables when the proportion of outliers was 10% or 15%.

In terms of variable selection, when there were a small proportion of outliers, Ensemble performed best. However, its accuracy was greatly decreased when the proportion of outliers was large. In terms of outlier detection, regardless of the portion of outliers, MTL-EN had the highest outlier detection accuracy among the three methods.

### 4.2. Combining with Ensemble to Improve the Accuracy of Variable Selection

In our previous study [9], we considered a two-step procedure when the proportion of outliers was relatively large. We found that it improved the variable selection accuracy by applying Ensemble on a subset with outliers identified by enetLTS removed. In this study, we also used MTL-EN to detect outliers and then applied Ensemble on the subset with outliers removed. The results of MTL-EN and enetLTS were compared by simulation, which is shown in Table 1.

From Table 1, compared with the results in the original data, the PSR of Ensemble raised from 0.533 to 0.644, and the GM was improved from 0.714 to 0.786 for subset after removing outliers identified by enetLTS. For subset with outliers identified by MTL-EN removed, the results of Ensemble were also improved with PSR increased from 0.533 to 0.708 and GM increased from 0.714 to 0.828. It can be seen that after removing the outliers identified by MTL-EN, the accuracy of Ensemble variable selection is the highest.

### 4.3. The Computation Times of enetLTS and MTL-EN

From Table 2, the computation time of enetLTS is 39 times that of MTL-EN (Intel Core i7-6500U @2.50GHz); that is, the computation time of MTL-EN was 2% of that of enetLTS. This is because the C-step algorithm used by enetLTS does not take into account the regularized parameters that need to be determined at each step of the iteration. The criterion function cannot be guaranteed to gradually decrease, which makes the algorithm converge slowly. The AR-Cstep algorithm adopted by MTL-EN solves this problem well, which greatly improves the convergence speed.

## 5. Case Study

In the previous study [9], we compared the application of enetLTS, Ensemble, and Rlogreg on a TNBC dataset from the TCGA-BRCA data collection. The results showed that enetLTS identified 68 outliers, seven of which were individuals with inconsistent labels. After removing the outliers identified by enetLTS, the prediction accuracy of the three Ensemble models was improved, and the number of associated genes identified increased from 5 to 9. In this study, we applied MTL-EN to this TNBC dataset. The outliers identified by MTL-EN were compared with those by enetLTS, and we also compared the performances of Ensemble after removing the outliers identified by MTL-EN and enetLTS, respectively.

From Tables 3 and 4, among the 68 outliers identified by enetLTS, 3 of them were labeled as TNBC, which were also identified by MTL-EN; among them, 65 individuals with non-TNBC labels included 35 non-TNBC patients identified by MTL-EN. In other words, 38 of the 47 outliers with non-TNBC labels identified by MTL-EN were also identified by enetLTS. However, nine patients with TNBC labels were not identified by enetLTS. These 9 TNBC patients were highly expressed in one or more of the three genes, suggesting that they were likely to be non-TNBC patients or misclassified individuals. For example, TCGA-BH-A42U (HER2 38.37), TCGA-E2-A1L7 (ER 29.61, PR 22.98), TCGA-OL-A97C (PR 8.56), TCGA-A2-A1G6 (ER 23.90, PR 21.45, HER2 29.74), TCGA-A2-A0EQ (ER 2.13, HER2 30.15), TCGA-EW-A1OV (HER2 28.91), TCGA-OL-A5D6 (HER2 72.13), TCGA-C8-A26X (HER2 60.12), and TCGA-LL-A740 (HER2 68.56), with high expression in one or more of three receptors, were more likely not to be a TNBC patients; that is, his/her labels were probably wrong. Seven of the 47 outliers identified by MTL-EN were suspect individuals with inconsistent HER2 labels. Six of them were labeled as non-TNBC, which were also detected by enetLTS. The remaining one “TCGA-A2-A0EQ” was labeled as TNBC, which was not detected by enetLTS.

A total of 213 genes were identified by MTL-EN, and 40 genes with the largest absolute value are listed in Table 5. Among them, FOXA1 [17], ERBB2 [18], GRB7 [19], KRT16 [20], CXXC5 [21], FOXC1 [22], TFF3 [23], COL9A3 [24], FABP7 [25], CCNE1 [26], GZMB [27], and MIEN1 [28] were reported to be related to TNBC.

In our previous study [9], we combined the advantages of enetLTS and Ensemble and removed 68 outliers identified by enetLTS, then ran Ensemble on a subset (856 samples), to improve the accuracy of gene selection. In this study, we removed 47 misclassification samples detected by MTL-EN and then ran Ensemble in the remaining 877 samples. The results are shown in Tables 6 and 7.

From Table 6, for the subset with outliers detected by enetLTS removed, the prediction index MR of the three models in Ensemble was much lower than that on the original TNBC dataset; the MR of EN decreased from 0.012 to 0, the SPLS-DA MR reduced from 0.064 to 0.008, and the SGPLS MR reduced from 0.059 to 0.015. When Ensemble was run on a subset of 47 outliers identified by MTL-EN, the prediction accuracy MR of the three models in Ensemble also decreased greatly, to 0.001, 0.014, and 0.013, respectively.

For subset with 68 outliers detected by enetLTS removed, the intersection of variables selected using the three Ensemble models increased from five to nine genes, namely, CA12 [29], GABRP [30], VGLL1 [31], AGR2 [32], GATA3 [17], FOXA1 [17], TFF3 [23], AGR3 [33], and KRT16 [20], were reported to be related to TNBC.

From Table 7, for subset with 47 outliers detected by MTL-EN removed, the intersection of variables selected using the three Ensemble models was 12 genes. Among them, ESR1, one of three key variables, and FOXC1 [22], AGR2 [32], FOXA1 [17], TFF3 [23], TFF1 [34], AGR3 [33], KRT6B [35], and KRT16 [20] have been reported to be related to TNBC. KLK6 [36], FDCSP [37], and PPP1R14C [38] have been reported to be related to other types of tumors. Their association with TNBC needs further study.

## 6. Discussion

Through our previous research [9], we have found that in high-dimensional data with mislabeled error, robust trimmed penalized regression is a recommended method in identifying mislabeled samples. However, the C-step algorithm to implement this method (enetLTS) is too slow to meet the requirement of data analysis for high-dimensional omics data. The reason is that for LTS without regularized parameters, the inequality that guarantees the convergence of the C-step algorithm is established. However, for the robust trimmed penalized regression with regularized parameters, the inequality does not necessarily hold due to the change of the regularized parameters.

In the AR-Cstep algorithm, penalized regression is repeatedly performed on the subset at each step to concentrate on the individuals who fit the model best gradually; that is, the idea of the C-step algorithm is still adopted. However, AR-Cstep can solve the problem of the C-step algorithm not converging because the regularized parameters change during the iteration. A comparison of the likelihood function of the current subset and that of the candidate subset is used to determine whether to replace the current subset with the candidate subset in AR-Cstep, thereby ensuring that the iterative process is in the direction that improves the criterion function. To avoid falling into a local optimum, the Metropolis-type probabilistic acceptance-rejection algorithm is combined.

Through simulation experiments, it is found that MTL-EN using AR-Cstep algorithm was more accurate than enetLTS using C-step algorithm in outlier identification. In particular, the accuracy of Ensemble variable selection on the subset after removing outliers identified by MTL-EN was higher than the result of Ensemble running on the subset after removing outliers identified by enetLTS. The AR-Cstep algorithm adopted by MTL-EN greatly improved the convergence speed; that is, the computation time of MTL-EN was 2% of that of enetLTS.

If a misclassified sample identified by a certain method is labeled as non-TNBC, it means that the expression of the key genes ER, PR, or HER2 is false positive in this patient. Similarly, if a misclassified sample identified is labeled as TNBC, it implies that the expression of ER, PR, or HER2 is a false negative in the patient. In the analysis of the TNBC dataset, there are 153 individuals labeled as TNBC in this TNBC dataset. There are 3 samples identified by enetLTS that were labeled as TNBC patients with false negative rate 2% (3/153). Twelve individuals labeled as TNBC patients were identified as mislabeled samples by MTL-EN with false negative rate 7.8% (12/153). In the TNBC dataset, IHC test of ER and PR was adopted for all patients. For HER2 detection, the results of IHC were for 507 patients. According to previous studies, the false negative rates of IHC test for ER, PR, and HER2 were not low, 15.1% ~21.8% for ER [39], 6.8% (4/58) for PR [40], and 6.2% (4/65) for HER2 [41], respectively. Therefore, the false negative misclassified samples identified by MTL-EN were more likely to be close to the reality than enetLTS.

A large class of computational problems in robust statistics can be formulated as the selection of the optimal subset of data based on some criterion function [10]. AR-Cstep algorithm, as the improvement of C-step algorithm, can be extended to other robust models with regularized parameters. It is an effective algorithm for finding the most suitable subset of regularized models, such as robust Adaptive LASSO, Group LASSO, SCAD, and MCP. The AR-Cstep algorithm can be extended to other generalized linear models, such as penalized multiclass logistic regression and penalized Poisson regression.

## 7. Conclusion

AR-Cstep can solve the problem of the C-step algorithm not converging because the regularized parameters change during the iteration. It provides an idea for developing the efficient algorithm of robust penalized regression based on trimming. The AR-Cstep algorithm can be extended to other robust models with regularized parameters. In practice, MTL-EN using AR-Cstep algorithm is the recommended method for mislabeled sample identification in omics data because of its high accuracy and high operation speed. When the proportion of mislabeled samples is relatively low and ≤5%, Ensemble can be used for variable selection. When the proportion of mislabeled samples is >5%, Ensemble can be used for variable selection on a subset of data after removing mislabeled samples identified by MTL-EN.

## Figures and Tables

**Figure 1:** Results of MTL-EN, enetLTS, and Ensemble when *n* = 500 and *p* = 1000. Sn: sensitivity; FPR: False Positive Rate; PSR: Positive Selection Rate; FDR: False Discovery Rate.

**Algorithm 1:** Description of C-step algorithm.

**Algorithm 2:** Description of AR-Cstep algorithm.

**Table 1:** Results of Ensemble for the datasets with *n* = 500, *p* = 1,000, and *ε* = 0.15.

Data	Model size	PSR	FDR	GM^#^
Original data	16.06	0.533	0.003	0.714
Subset^∗^	19.79	0.644	0.022	0.786
Subset^∗∗^	21.75	0.708	0.021	0.828

^∗^This subset is the original dataset after removing outliers identified by enetLTS. ^∗∗^This subset is the original dataset after removing outliers identified by MTL-EN. #*G*M: the geometric mean of PSR and (1-FDR).

**Table 2:** Computation times of MTL-EN and enetLTS for the datasets with *n* = 500, *p* = 1,000, and *ε* = 0.1.

Methods	Mean(s)
enetLTS	6489.06
MTL-EN	165.2

**Table 3:** Number of misclassified observation that detected using enetLTS and Ensemble.

Method	Identified misclassification	Num of TNBC/non-TNBC^∗^	Num of suspect TNBC/non-TNBC^∗∗^
enetLTS	68	3/65	0/7
MTL-EN	47	12/35	1/6

^∗^Number of identified misclassified observations with TNBC/non-TNBC labels. ^∗∗^Number of identified suspect individuals with inconsistent labels.

**Table 4:** Forty-seven misclassified observations detected using MTL-EN for the TNBC dataset^#^.

ID	ESR	PGR	HER2	HER2_level	HER2_status	HER2_FISH	*y*	Perres
TCGA-E9-A22G	0.44 (-)	0.02 (-)	15.32		+		Non-TNBC	32.54
TCGA-A2-A3Y0	2.18 (+)	0.03 (-)	11.34	1+	-		Non-TNBC	29.71
TCGA-A2-A04U	0.02 (-)	0.02 (-)	9.64	1+	-	+	Non-TNBC	22.86
TCGA-BH-A1EW	29.98 (-)	18.90 (-)	42.47		-		TNBC	18.89
TCGA-GM-A2DI	23.49 (-)	12.05 (-)	20.30			-	TNBC	14.73
TCGA-S3-AA0Z	16.67 (+)	0.07 (+)	33.07	1+	Equiv	-	Non-TNBC	14.58
TCGA-AN-A0FJ	0.08 (+)	0.04 (-)	14.28	1+	+		Non-TNBC	14.03
TCGA-BH-A5IZ	5.12 (+)	0.03 (-)	28.08		-	-	Non-TNBC	13.87
TCGA-OL-A5S0	0.09 (+)	0.06 (-)	31.92			+	Non-TNBC	13.45
TCGA-E9-A1ND	1.44 (-)	0.05 (-)	13.05		+		Non-TNBC	13.05
TCGA-B6-A0IJ	1.18 (+)	0.46 (+)	11.12				Non-TNBC	11.92
TCGA-AR-A251	1.57 (+)	0.10 (-)	14.02	2+	Equiv	-	Non-TNBC	10.70
TCGA-D8-A1JM	5.00 (+)	0.01 (-)	21.85	1+	-		Non-TNBC	10.52
TCGA-E2-A1II	0.14 (-)	0.19 (+)	10.73	1+	-		Non-TNBC	10.51
TCGA-A2-A1G6^∗^	23.90 (-)	21.45 (-)	29.74	1+	-		TNBC	9.62
TCGA-A2-A0YJ	0.09 (+)	0.03 (-)	240.24	0	-		Non-TNBC	9.52
TCGA-LL-A5YP	0.16 (+)	0.05 (-)	15.10	1+	-	+	Non-TNBC	9.23
TCGA-E9-A1NC	0.11 (-)	0.07 (+)	15.91		+		Non-TNBC	8.98
TCGA-AC-A62X	0.19 (+)	0.02 (-)	28.53				Non-TNBC	8.93
TCGA-A7-A13E	0.82 (+)	0.06 (-)	46.08	2+	Equiv	-	Non-TNBC	8.77
TCGA-C8-A3M7	4.27 (-)	0.76 (-)	25.47		-		TNBC	8.71
TCGA-AR-A1AJ	1.47 (+)	0.07 (-)	9.74		-		Non-TNBC	8.53
TCGA-BH-A0DL	6.99 (+)	0.04 (-)	9.92		-		Non-TNBC	7.85
TCGA-E2-A1L7^∗^	29.61 (-)	22.98 (-)	10.33		-		TNBC	7.35
TCGA-AR-A1AH	0.03 (+)	0.03 (-)	34.12		-		Non-TNBC	7.31
TCGA-E2-A14Y	0.67 (+)	0.03 (+)	487.90	2+	Equiv	+	Non-TNBC	7.11
TCGA-LL-A8F5	1.08 (+)	0.04 (-)	11.86	1+	-		Non-TNBC	6.96
TCGA-OL-A97C^∗^	16.25 (-)	8.56 (-)	24.04			-	TNBC	6.86
TCGA-A7-A13D	0.52 (-)	0.81 (+)	42.28	2+	Equiv	-	Non-TNBC	6.73
TCGA-AR-A0TP	0.04 (+)	0.03 (-)	13.39		-		Non-TNBC	6.53
TCGA-LL-A6FR	0.33 (-)	0.04 (+)	32.13	2+	Equiv	+	Non-TNBC	6.19
TCGA-A2-A25F	0.62 (-)	0.23 (+)	5.19		-		Non-TNBC	5.86
TCGA-AO-A0JL	0.63 (-)	0.08 (-)	63.60	1+	-	+	Non-TNBC	5.45
TCGA-A2-A1G1	0.53 (-)	0.17 (-)	819.76	2+	Equiv	+	Non-TNBC	5.28
TCGA-BH-A42U^∗^	9.19 (-)	1.83 (-)	38.37		-		TNBC	4.99
TCGA-AN-A0FX	1.13 (-)	0.64 (-)	24.02	1+	+		Non-TNBC	4.75
TCGA-D8-A1XW	0.32 (-)	0.11 (+)	21.03	1+	-		Non-TNBC	4.57
TCGA-AR-A24Q	1.00 (+)	0.36 (-)	20.67		-		Non-TNBC	4.52
TCGA-A1-A0SB	3.16 (+)	0.03 (-)	32.35		-		Non-TNBC	4.47
TCGA-A2-A4RX	0.68 (+)	0.93 (+)	26.64	1+	-		Non-TNBC	3.18
TCGA-AN-A0FL	0.09 (-)	1.07 (-)	15.07	1+	+		Non-TNBC	3.01
TCGA-A2-A0EQ^∗^	2.13 (-)	0.04 (-)	30.15	3+	+	-	TNBC	2.63
TCGA-EW-A1OV^∗^	0.23 (-)	0.03 (-)	28.91		-	-	TNBC	1.83
TCGA-OL-A5D6^∗^	0.35 (-)	0.20 (-)	72.13			-	TNBC	1.69
TCGA-C8-A26X^∗^	0.42 (-)	0.13 (-)	60.12	1+	-		TNBC	1.62
TCGA-LL-A740^∗^	0.30 (-)	0.12 (-)	68.56	2+	Equiv	-	TNBC	1.48
TCGA-BH-A6R9	0.59 (-)	0.25 (+)	8.18		-		Non-TNBC	0.99

#Including the expression values, IHC, and FISH tests of ER, PR, and HER2 (individuals highlighted in bold are suspect individuals). ^∗^Outliers detected by MTL-EN but not by enetLTS. ^∗∗^Perres: the abstract value of Pearson residual.

**Table 5:** Top 40 genes selected by MTL-EN for the TNBC dataset.

Upregulated	COX7B2 (0.14), LBP (0.12), SLC15A1 (0.11), B3GNT5 (0.10), A2ML1 (0.10), FOXC1 (0.09), COL9A3 (0.09), KRT16 (0.09), FDCSP (0.09), FABP7 (0.09), AADAT (0.09), VSNL1 (0.09), KLK6 (0.09), PPP1R14C (0.08), GZMB (0.07), CCNE1 (0.07), FAM171A1 (0.07)
Downregulted	AGR3 (-0.24), CA12 (-0.20), AGR2 (-0.19), MLPH (-0.17), ESR1 (-0.15), TBC1D9 (-0.13), FOXA1 (-0.12), TFF1 (-0.12), ERBB2 (-0.11), GRB7 (-0.10), STARD3 (-0.10), PGAP3 (-0.10), TFF3 (-0.10), CXXC5 (-0.10), GATA3 (-0.10), ACOX2 (-0.09), ASPN (-0.09), MIEN1 (-0.08), SPDEF (-0.08), CHAD (-0.08), EEF1A2 (-0.08), CMBL (-0.08), SRARP (-0.07)

**Table 6:** Results of Ensemble three models for the original TNBC data and subset with outliers removed.

Dataset	EN		SPLS-DA		SGPLS	
	Model size^∗∗^	MR^#^	Model size	MR	Model size	MR
Original data	175	0.012	22	0.064	33	0.059
Subset^∗^	83	0.000	87	0.008	16	0.015
Subset^##^	49	0.001	38	0.014	55	0.013

^∗^This subset is the original dataset after removing 68 outliers identified by enetLTS. ##This subset is the original dataset after removing 47 outliers identified by MTL-EN. ^∗∗^Model size: number of variables; #MR: misclassification rate.

**Table 7:** Genes selected by Ensemble for the TNBC subset^∗^.

FOXC1, ESR1, AGR2, FOXA1, TFF3, TFF1, KLK6, AGR3, FDCSP, KRT6B, KRT16, PPP1R14C

^∗^This subset is the original dataset after removing 47 outliers identified by MTL-EN.

## Data Availability

Code is available on Github (https://github.com/hwsun2000/AR-Cstep). The BRCA RNA-Seq FPKM dataset was imported using the “brca.data” R package (https://github.com/averissimo/brca.data/releases/download/1.0/brca.data_1.0.tar.gz).
